# Cost-Effectiveness of Oral Antidiabetic Drugs: A Prospective Multicenter Study of Real-World Patients

**DOI:** 10.1155/2021/9972386

**Published:** 2021-10-28

**Authors:** Gordon Liu, Zhiyong Huang, Qian Xin

**Affiliations:** ^1^Institute for Global Health and Development, Peking University, Beijing 100871, China; ^2^Center of Health Policy and Governance, Southwestern University of Finance and Economics, Chengdu 611130, China; ^3^Visible Analytics, Oxford OX20DP, UK

## Abstract

This real-world, multicenter, prospective study aims to analyze the cost-effectiveness of prevalent oral antidiabetic drugs, including traditional Chinese medicine and its compounds, used in China. Type 2 diabetes patients initiated on one or several of the most prevalent antidiabetic drugs were recruited on the baseline and followed up over one year with no restriction on drug discontinuation, switching, and add-on. Different drugs were evaluated on their efficacy, adverse effect (AE), health-related quality of life (HRQoL), and cost. Treatments were defined as the intent-to-treat in the primary analysis and on-treatment in the sensitivity analyses. A rich set of patients' baseline characteristics was collected and controlled using the multivariate linear model in the primary analysis and inverse probability weighting and double selection—a machine learning algorithm—in the sensitivity analyses. Estimates of “raw” outcomes, which are not adjusted by covariates and calculated as subgroup means, show that the use of Xiaoke Pill alone and in combination is among the most effective therapies with 50% and 54% of patients reaching the control target of HbA1c < 6.5%. In terms of cost, Xiaoke Pill and gliclazide, which cost participants 4,350 and 5,150 RMB per year on average, are among the least costly therapies. After adjusting patient characteristics, monotherapy and combination therapy using the Xiaoke Pill again display the best control rates, of 45% and 43% against 33% of metformin. Regarding cost, the Xiaoke Pill costs a patient 5,340 RMB per year, in sharp contrast with 8,550 RMB for metformin and 10,330 RMB for acarbose. Our study suggests that the use of Xiaoke Pill—alone or in combination—is associated with better glycemic control and lower cost than some allopathic medications such as metformin or acarbose and shows a similar incidence of hypoglycemia.

## 1. Introduction

In 2019, 463 million adults (one in 11 adults) aged between 20 and 79 years had diabetes mellitus worldwide, and the number is projected to reach 578 million by 2030 and 700 million by 2045 [1]. The high prevalence of diabetes represents huge health and economic burdens. In 2016, diabetes caused 1.599 million deaths, which ranked it the seventh leading cause of death [2]. In 2019, an estimated $ 760 billion was spent on diabetes treatment, making up 10% of the global health expenditure spent on adults [1]. With the rising prevalence of diabetes globally, low- and middle-income countries have experienced the greatest increase in recent years [1]. In China, an estimated 129.8 million adults have diabetes, which accounts for 11.2% of its adult population [3], and the health expenditure attributed to diabetes was estimated to be $ 63 billion [1].

In China, diabetes is treated with both allopathic medicines and traditional Chinese medicine (TCM). The history of using TCMs as a treatment for diabetes is over 2000 years [4]. Nowadays, many of the TCMs have been included in the national reimbursement plan and TCM alone or in combination with allopathic drugs has been widely prescribed in clinical settings [5]. A survey conducted at 75 hospitals in nine cities found that the proportions of patients treated with biguanides, sulfonylurea, meglitinides, glitazones, *α*-glucosidase inhibitors, and others (including TCMs) were 78.4%, 65.1%, 14.0%, 12.6%, 31.1%, and 18.1%, respectively. Oral antidiabetic drugs on 2018 China's National Essential Medicines, which is the most recently issued guidance for purchase and reimbursement of essential drugs by healthcare providers in China, include both allopathic drugs, such as metformin, glibenclamide, glipizide, glimepiride, gliquidone, gliclazide, acarbose, dapagliflozin, liraglutide, repaglinide, pioglitazone, sitagliptin, and linagliptin, and TCMs, such as the Xiaoke Pill (*Xiao Ke Wan* in Chinese).

Among TCMs used in treating diabetes, the Xiaoke Pill, a compound of glibenclamide and several Chinese herbs, was widely used to treat diabetes in China [6]. The Xiaoke Pill contains 0.25 micrograms of glibenclamide (per pill) and Chinese herbs such as Radix Puerariae, Radix Rehmanniae, Radix Astragali, Radix Trichosanthis, Stylus Zeae Maydis, Fructus Schisandrae Sphenantherae, and Rhizoma Dioscoreae, selected according to two ancient TCM formulas, namely, “Yuquan San” and “Xiaoke Fang.” An experiment using rats showed that Radix Astragali, one of the TCM substances of the Xiaoke Pill, could amplify the glucose counterregulatory response to insulin-induced hypoglycemia [7]. A randomized, double-blind, and multicenter clinical trial found that the Xiaoke Pill, compared with glibenclamide, had similar glucose control efficacy but a reduced risk of hypoglycemia, which indicated that TCM herbs in the Xiaoke Pill were protective against hypoglycemia caused by glibenclamide [8].

Given the high prevalence and economic burden of diabetes, studies on the cost-effectiveness of antidiabetic drugs are needed to plan treatment programs. One previous study, which compared five oral antidiabetic drugs in the Chinese market, found that metformin was cost-effective [9]. Another study found metformin to be cost-effective against acarbose [10]. However, a systematic review of 16 cost-effectiveness studies conducted in China found that metformin was the least cost-effective therapy when compared to rosiglitazone, glipizide, and *α*-glucosidase inhibitors [11]. There are some other studies regarding the cost-effectiveness of antidiabetic drugs other than metformin in China [12]. However, most of the existing studies on the cost-effectiveness of antidiabetic drugs used in the Chinese market are limited by their relatively small sample sizes, retrospective or model-based designs, and lack of information on the actual cost undertaken by patients.

In this study, we aim to analyze the cost-effectiveness of currently existing oral antidiabetic drugs in the management of type 2 diabetes in China, including TCMs and TCM compounds. In particular, we compare the efficacy, adverse effect, HRQoL, and cost among the most commonly used oral antidiabetic drugs in China with real-world evidence. We contribute to the existing literature in several ways. First, the cost-effectiveness studies of oral antidiabetic drugs in the Chinese market are lacking, especially for TCMs, although TCMs are routinely used for diabetes treatment. In this study, we analyze the cost-effectiveness of TCMs and their compounds, among other commonly used antidiabetic drugs. Second, the real-world design of this study can help us better assess the cost-effectiveness of different types of diabetes therapies in medical practice where discontinuation, switching, and add-on behaviors are common but difficult to incorporate into the model-based analysis. Third, our study is of multicenter and prospective design and of a relatively large size, providing us with enough statistical power to capture significant differences in key outcomes of interest.

As a complementary source to conventional randomized controlled trials (RCTs), real-world evidence has become increasingly important in healthcare decision-making [13]. Cost-effectiveness analysis based on real-world evidence has advantages, such as focusing on effectiveness rather than efficacy, simultaneous comparison of multiple treatment options, and rich data on resource use, but confounding bias associated with real-world data should be addressed with great caution [14]. To date, there have been very few real-world studies on the cost-effectiveness of antidiabetic drugs. A retrospective study compared liraglutide with exenatide, in which the multivariate regression was used to control confounding bias [15]. Another retrospective study compared canagliflozin with dapagliflozin, in which the propensity score-based method was used to adjust the confounding bias [16]. In this study, we adopted a prospective, observational cohort design [14] and collected a wide range of potential confounding factors of health outcomes and costs associated with diabetes, following a systematic review of the existing evidence. During the analysis stage, several statistical methods, including multivariate regression, inverse probability weighting, and double selection, were used to mitigate confounding bias.

## 2. Materials and Methods

### 2.1. Study Design and Sample

This study was a prospective multicenter study of real-world patients. The Ethics Review Committee of The Third Affiliated Hospital of Peking University of Traditional Chinese and Western Medicine approved the study. All the participants provided their written informed consent to participate in this study. Participants were recruited from 66 community health centers located in five Chinese cities (i.e., Beijing, Chengdu, Guangzhou, Nanjing, and Shenyang) between December 2010 and December 2011. Recruitment was facilitated by an endocrinologist (or a general practitioner if the health center did not have an endocrine department) and was assisted by trained interviewers. All clinically diagnosed patients with type 2 diabetes who visited the healthcare centers in 2010 and provided phone numbers were contacted and screened for eligibility for inclusion. (1) Patients aged 16 years or older who were clinically diagnosed with type 2 diabetes; (2) those who were taking oral antidiabetic drugs, without any cognitive impairment, severe vision problems, or hearing problems; (3) those who were able to read and communicate in Mandarin; and (4) those who were willing to participate in the study were considered eligible. Among all eligible patients, 3,000 subjects (with a target of 600 in each city) were randomly sampled with a quota of 600 subjects for users of the Xiaoke Pill.

Upon completing the baseline interview, the patients were invited to participate in follow-up surveys every three months, four times per year. In addition, two medical tests were administrated, one at the time of the baseline interview and the other at the last follow-up, to collect physiological indicators associated with patients' diabetic conditions.

A number of quality control measures were taken throughout the survey. First, a pilot test was conducted before the baseline survey to test the survey design. Second, both investigators and supervisors were screened and trained. Investigators were recruited from our cooperators, including Beijing University of Chinese Medicine in Beijing, Shenyang Pharmaceutical University in Shenyang, China Pharmaceutical University in Nanjing, Southwestern University of Finance and Economics in Chengdu, and Guangzhou Academy of Social Sciences in Guangzhou, while supervisors were recruited from the China Center of Health Economics Research. A survey guide was provided to both investigators and supervisors. Third, every filled questionnaire was checked by two reviewers independently. Fourth, 20% of filled questionnaires were randomly selected and called back by phone. Last, a double-entry method was adopted to ensure the accuracy of data entry.

In the statistical analysis stage, we kept those who had participated in the baseline, all follow-up surveys, and the two medical tests. We excluded those taking insulin at the baseline but imposed no restriction on initial oral drug use, following discontinuation, switching, and add-on of drugs (Figure 1). There were 1903 subjects remaining in our working sample, with 440 from Shenyang, 314 from Beijing, 403 from Chengdu, 366 from Nanjing, and 380 from Guangzhou. The power of results from each city might not be even due to differences in sample sizes. However, there were enough observations for each city so that meaningful inference can be reached.

### 2.2. Measures

Table 1 describes the variables of outcomes, treatments, and controls used in this study.

#### 2.2.1. Outcomes

We evaluated the outcome of each drug in terms of its efficacy, AE, HRQoL, and associated costs, including hospitalizations, outpatient encounters, and OTC pharmacy prescriptions. Note that hospitalizations include the expense for drugs used in the episode of inpatient care and outpatient encounters include the expense for drugs in the episode of outpatient care.

*(1) Efficacy*. Efficacy was measured as the level of glycemic control with the glycated hemoglobin (HbA1c) target of <6.5% recommended by the American Diabetes Association, the European Association for the Study of Diabetes, the International Diabetes Federation, and the WHO [17]. The indicator variable takes the value of one under control target or zero out of control target.

*(2) AE*. As a side effect associated with antidiabetic drugs, hypoglycemia (also known as low blood sugar) is considered a major AE concern in diabetes treatment. This study asked patients whether they had experienced hypoglycemia since the last survey. If they had, the AE indicator was coded as one and if not, zero during that period. The AE measure was then calculated as the sum of the AE indicators over the four follow-up surveys and ranged from zero to four.

*(3) HRQoL*. Patients were asked to complete an EQ-5D-3L questionnaire at baseline and follow-up surveys [18]. Answers to these questions were transformed into HRQoL scores using the value set for the Chinese population [19]. The HRQoL score is defined as a continuous measure ranging between zero and one.

*(4) Costs*. Given our real-world setup, we measured the all-cause medical costs incurred to diabetic patients without making a distinction between costs directly attributable to diabetes and other indirect medical costs [20]. We measured the costs of the inpatient and outpatient services (including the cost of drugs prescribed and purchased within hospitals and clinics), as well as OTC drug costs. The total cost was defined as the sum of inpatient cost, outpatient cost, and OTC drug costs.

#### 2.2.2. Treatment

In this real-world study, we monitored the use of up to 15 different types of oral antidiabetic medications, including biguanides (metformin and phenformin), sulfonylureas (glibenclamide, glipizide, gliquidone, gliclazide, and glimepiride), *α*-glucosidase inhibitors (acarbose and voglibose), secretagogue (repaglinide and nateglinide), thiazolidinediones (rosiglitazone and pioglitazone), TCMs, and the Xiaoke Pill. No restriction on drug use behaviors such as discontinuation, switching, and add-on of drugs was imposed. Using this design, we could observe a pyramid of therapies for diabetes adopted in medical practice. To maintain sufficient statistical power, we restrict our analysis on several drugs most widely used.

In this study, we focus on intent-to-treat (ITT), defined as therapies chosen by patients at the time of the baseline survey [21]. At baseline, we observed 132 different plans, including monotherapies and combination therapies among patients. We kept the top five monotherapies with the largest proportions of users but also glibenclamide, which constituted one important substance of the Xiaoke Pill. In addition, we included a combination therapy of the Xiaoke Pill. All other therapies were merged into the category of “others” for comparison. Therefore, our ITT treatment variable was defined as a categorical variable representing the eight therapies. The number of patients in each therapy group is summarized in Table 2. Metformin and the Xiaoke Pill accounted for 10.67% and 12.24%, respectively, while another 9.3% of patients used the Xiaoke Pill in combination with other drugs. Complete descriptions of the composition of all therapies in our sample are listed in Table 3.

In addition to the estimates of ITT, we estimated the on-treatment effect by only including patients who adhered to the same therapy without discontinuation, switching, or add-on of drugs throughout the study. Although the on-treatment effect could avoid the “dilution effect” caused by dropping out and switching, it is criticized for reduced sample size and bias due to using only compliers [22]. Analysis of the on-treatment effect was included in the sensitivity analyses.

#### 2.2.3. Covariates

To reduce confounding bias, we collected and controlled a rich set of individual baseline characteristics of survey patients, which was crucial to real-world analysis to recover the treatment effect. We controlled factors such as demographics including age and sex; socioeconomic factors including education, household income, type of medical insurance, and city of residence; diabetes-related morbidities including heart disease, hypertension, dyslipidemia, and stroke; duration of diabetes; behavior factors including alcoholic use, smoking, physical exercise, and diet control; hypoglycemia as the primary adverse effect; anthropometric and physiological indicators including body mass index (BMI), fasting blood sugar level (FBS), HbA1c, systolic blood pressure (SBP), diastolic blood pressure (DBP), total cholesterol (TC), triglycerides (TG), and HRQoL measured as EQ-5D scores. All covariates were measured at the time of the baseline survey. BMI, FBS, HbA1c, TC, and TG were coded as dichotomous variables with clinically relevant cutoffs [17, 23, 24]. The descriptive statistics of covariates by therapies are shown in Table 4 with the last column including significant levels derived from ANOVA tests regarding variance among different therapies. Most characteristics were imbalanced among different therapies at conventionally significant levels.

### 2.3. Statistical Methods

Similar to other observational studies, we imposed conditional independence (CI) to identify treatment effects among different therapies [25]. The CI assumption says that, after conditioning on covariates, the treatment variable is independent of the outcome variable. The CI assumption is justified by the rich set of covariates we have controlled for. In addition to this crucial assumption, we have some other model-specific assumptions, which we illustrate in the following.

#### 2.3.1. Multivariate Linear Regression

In our primary analysis, we used multivariate linear regression to estimate the treatment effects of drugs. The multivariate linear regression has the advantage of establishing meaningful inference when some treatment arms have very few observations. It is helpful for our study since one treatment arm in our study, glibenclamide, has few observations, precluding us from implementing data-driven statistical models. The disadvantage of multivariate linear regression is that it relies on the correct specification of functional forms. We addressed this potential problem in the sensitivity analysis, in which the propensity score-based method and machine learning methods were used for comparison.

#### 2.3.2. Inverse Probability Weighting

As an alternative to multivariate regression, the inverse treatment assignment as weights is widely used to estimate treatment effects with multiple treatment arms [26–28]. Note that there are some other popular propensity score-based methods such as matching, stratification, and imputation, which, however, are hard to be implemented on studies with many treatment arms like ours. Inverse probability weighting (IPW) reduces confounding bias by reweighting treatment arms to mimic a random assignment, in which the weights are typically calculated as the functions of propensity score defined as the probability of receiving treatment conditional on covariates [29]. The IPW is less susceptible to functional misspecification; however, it requires more data than regression models. In this study, we used multinomial logistic regression to obtain the propensity score of each treatment arm.

#### 2.3.3. A Machine Learning Algorithm: Double Selection Lasso on High-Dimensional Control Variables

Including a large set of covariates can help minimize confounding bias, but it has the cost of the reduced efficiency of estimation, as it inflates both the signal and noise. The least absolute shrinkage and selection operator (lasso) [30] and its variations such as adaptive lasso [31] have been widely used to select covariates in high-dimensional models in the context of prediction. However, designed for prediction, not for causal inference, lasso and adaptive lasso are likely to produce an unreliable estimate for the treatment effect [32], which is the central goal of our study. Recently, some lasso-like estimators were proposed to make causal inference in a high-dimensional model [33–35]. In this study, we used a double selection lasso estimator to estimate treatment effects [33, 34]. First, we created a pool of potential covariates, including the variables listed in Table 1 and their interaction terms. Note that, technically, we also included squared terms of these variables but they were identical to the original variables which were defined as dummies. After dropping the variables with collinearity, we were left with 69 covariates. We then used the adaptive lasso method to select covariates for the outcome and treatments. Finally, we operated multivariate regressions using the union of selected covariates for the outcome and treatments as control variables. The detailed algorithm is displayed in Appendix.

## 3. Results

### 3.1. Unadjusted Outcomes on Effects and Costs

Estimates of “raw” outcomes that are not adjusted by covariates are calculated as subgroup means (Figures 2 and 3). Results of pairwise tests among different therapies are included in Table 5, where the estimates sharing a letter in the group label are not significantly different at the 5% level.

In terms of glycemic control, the use of the Xiaoke Pill alone and in combination was among the most effective therapies, with 50% and 54% of patients reaching the control target of HbA1c level <6.5%, respectively. At the conventional statistical level, the effects were significantly different for metformin (with a control rate of 33%). On the other hand, TCMs other than Xiaoke Pill had the lowest control rate, with only 20% of the patients having attained the control target.

In terms of AE measured as the incidence of hypoglycemia, patients using the Xiaoke Pill in combination with other drugs experienced the least number of adverse events, with the incidence of 0.27 times in one year on average, while TCMs other than Xiaoke Pill had the highest reported occurrence of low-blood-sugar events, 0.72 times per year. No significant difference was found among other therapies, including the use of the Xiaoke Pill alone or metformin alone. The HRQoL difference among different therapies was relatively marginal although the Xiaoke Pill and metformin show statistically significant higher uses.

Regarding the total cost, defined as the sum of costs of inpatient and outpatient care, and OTC drugs, the Xiaoke Pill and gliclazide, which cost participants 4,350 (around $670) and 5,150 RMB per year on average, are among the least costly therapies (significantly lower than other therapies at the 5% significance level). Note that even with the lowest point estimate of the cost, the cost of glibenclamide is not statistically lower than other plans in our analysis. The most expensive therapy is acarbose which users, on average, need to spend 11,370 RMB in one year.

### 3.2. Adjusted Outcomes on Effects and Costs: Intent-to-Treat Treatment Effect

Table 6 provides a point estimate of treatment effects of different therapies with covariates adjusted using multivariate linear regressions. The use of the Xiaoke Pill alone and its combination with other drugs revealed superior effects, with control rates of 12% and 10% higher than those of the reference group of metformin, respectively, and the differences are significant at conventional levels. No statistically significant differences are found among drugs in terms of incidence of hypoglycemia, and the Xiaoke Pill in combination with other drugs shows slightly lower HRQoL than metformin. Regarding costs, compared with metformin, the Xiaoke Pill has significantly lower inpatient costs, acarbose displays higher outpatient costs, and TCMs and acarbose also show higher OTC drug costs. When considering the total cost, the cost reduction of the Xiaoke Pill against metformin is large and statistically significant.

To better understand the size of estimated treatment effects and make comparisons among all therapies rather than just contrasting one therapy with the reference drug, which is, in our case, metformin, we have calculated, in addition to the point estimates, the predictive margins. These are defined as predictive outcomes by fixing the treatment variable and averaging over covariates after regression. Note that the predictive margins for each treatment without covariates are just subgroup means. Therefore, predictive margins are comparable with subgroup means in the above analysis. The results of predictive margins are shown in Table 7 and Figures 4 and 5, respectively. In terms of glycemic control, monotherapy and combination therapy using the Xiaoke Pill again display the best control rates, of 45% and 43%, respectively, against 33% of metformin. However, the difference became smaller in comparison with the unadjusted outcomes, as shown in Table 5. The Xiaoke Pill costs a patient 5,340 RMB per year, in sharp contrast with 8,550 RMB for metformin and 10,330 RMB for acarbose. Although being lower than the unadjusted results, the cost difference among different therapies is still remarkable and statistically significant.

### 3.3. Sensitivity Analysis

Sensitivity analyses using a more conservative definition for treatment samples and more data-driven statistical methods such as inverse probability weighting and machine learning have provided consistent results on the effectiveness and cost of antidiabetic therapies. The detailed estimates are included in Appendix.

## 4. Discussion

Our study is one of the few studies that explore the cost-effectiveness of oral antidiabetic therapies, including TCM and its compounds, based on real-world evidence.

Our results show that metformin underperforms some other widely used antidiabetic drugs, including gliclazide and Xiaoke Pill, in terms of efficacy and cost. However, it has a lower incidence of adverse effects. This finding is consistent with some other studies. One meta-study found that thiazolidinediones, metformin, sulfonylureas, dipeptidyl peptidase-4 (DPP-4) inhibitors, and sodium-glucose cotransporter 2 inhibitors have similar efficacy [36]. Another study found that rosiglitazone, as compared with metformin, is associated with more extended glycemic durability from a clinical trial [37].

Our study provides some suggestive evidence that the Xiaoke Pill, as a compound formula of glibenclamide and Xiaoke herbal substance, may achieve better glycemic control than glibenclamide. However, the difference is not statistically significant given the small sample size of glibenclamide in our study. Our finding is consistent with a clinical trial [8], which evidenced that the Xiaoke Pill had either a similar or better effect in treating hyperglycemia in diabetic patients than glibenclamide. The benefit of the Xiaoke Pill may be linked to its Xiaoke herbs. It has been reported that the Xiaoke Pill not only exerts its antidiabetic activity by stimulation of insulin secretion mainly mediated by glibenclamide but also enhances the sensitivity of receptors towards insulin mediated by promoting adiponectin secretion in patients with diabetes [38]. Another study shows that several DPP-4 inhibitors are screened in the Xiaoke herbal substance [39].

Regarding add-on effects, our study suggests that the Xiaoke Pill added to metformin results in higher efficacy and lower incidence of AE. Another study also showed that DPP-4 on top of prior metformin monotherapy results in similar HbA1c reductions within 12 months but a significant reduction in hypoglycemia compared with sulfonylurea added to metformin [40].

Our study had several limitations of our study. First, we did not impose any restrictions on initiation, discontinuation, switching, and add-on of drug use, and we, therefore, had many different therapies used as treatments in our sample. Although with a relatively large sample, some treatment arms may not have enough observations to make meaningful statistical inference owing to the lack of power. Second, while we have included many baseline characteristics of patients as control variables, we may still have the omission of variables—a commonly criticized problem for all real-world studies. To address this concern, in sensitivity analyses, we utilize lasso to preselect a set of control variables from an extensive list of variables, including all baseline characteristics and their squared and interaction terms, and our conclusion is essentially the same. Third, our indicators on adverse effects are not complete in the sense that we did not include outcomes of risk of CVD and mortality [41]. However, including these outcomes require a much longer follow-up than is designed in this study.

Finally, it is worth noticing that it has been ten years since the data were collected and this lag may render some change on the cost of drugs and may undermine the validity of our results. Nevertheless, hopefully, readers may still find our study useful and relevant given the scant real-world evidence on the cost-effectiveness of antidiabetic drugs so far. Besides, we are assured by some aspects of our study, making our results less sensitive to this time lag. First, our analysis on efficacy and adverse events is unlikely to be biased by this time lag. Second, inpatient and outpatient costs are mainly driven by the efficacy, side effects, and quality of life change and thus less likely to be affected. In contrast, OTC medication cost, which is more subject to time change, accounts for relatively a small part of the total cost (23%). The last thing we want to emphasize is that even though ten years have passed, there are still minimal cost-effectiveness studies on antidiabetic drugs based on real-world evidence. We hope our study can generate some interest of researchers in this topic as it is very important for policy-making given the large and growing diabetes population in China.

## 5. Conclusions

Our study suggests that the use of Xiaoke Pill—alone or in combination—is associated with better glycemic control and lower cost than some allopathic medications such as metformin and shows a similar incidence of hypoglycemia.

## Figures and Tables

**Figure 1:** Study sample.

**Figure 2:** Unadjusted outcomes: efficacy, AE, and HRQoL. Note: point estimates of subgroup means and their 95% confidence intervals are drawn as circles and spikes. Dashed lines represent estimates of population means. Xiaoke Pill + refers to the use of Xiaoke Pill in combination with other antidiabetic drugs. (a) HbA1c < 6.5%. (b) Hypoglycemia. (c) EQ-5D.

**Figure 3:** Unadjusted outcomes: costs. Note: point estimates of subgroup means and their 95% confidence intervals are drawn as circles and spikes. Dashed lines represent estimates of population means. Xiaoke Pill + refers to the use of Xiaoke Pill in combination with other antidiabetic drugs. (a) Inpatient cost. (b) Outpatient cost. (c) OTC drug cost. (d) Total cost.

**Figure 4:** Risk factor-adjusted outcomes: efficacy, AE, and HRQoL. (a) HbA1c < 6.5%. (b) Hypoglycemia. (c) EQ-5D.

**Figure 5:** Risk factor-adjusted outcomes: costs. (a) Inpatient cost. (b) Outpatient cost. (c) Drug cost. (d) Total cost.

**Figure 6:** Risk factor-adjusted outcomes: efficacy, AE, HRQoL, and cost.

**Figure 7:** Inverse-probability-weighted outcomes.

**Figure 8:** Double selection.

**Table 1:** Description of variables.

Variables	Description
*Outcomes*	
HbA1c < 6.5%	1 if HbA1c < 6.5% at the last follow-up; 0 otherwise
Inci. of hypoglycemia	Incidence of reported hypoglycemia in one year (spanning the period of all four follow-up surveys)
EQ-5D HRQoL	HRQoL measured through EQ-5D
Inpatient cost	Inpatient cost in one year, including all costs related to tests, medication, and treatment in hospitals (unit: 1000 yuan)
Outpatient cost	Outpatient cost in one year, including all costs related to tests, medication, and treatment in clinics (unit: 1000 yuan)
OTC drug cost	OTC drug cost in one year (unit: 1000 yuan)
Total cost	Inpatient cost + outpatient cost + OTC drug cost (unit: 1000 yuan)

*Treatments*	
Metformin	Use of metformin alone
Xiaoke Pill	Use of Xiaoke Pill alone
TCMs	Use of other TCMs (with no chemical substance, other than Xiaoke Pill) alone
Gliclazide	Use of gliclazide alone
Acarbose	Use of acarbose alone
Xiaoke Pill+	Use of Xiaoke Pill in combination with other agents
Glibenclamide	Use of glibenclamide alone
Others	All other medication therapies

*Control variables*	
Age	Age categories: 1, younger than 50 (reference group); 2, aged between 50 and 60; 3, aged between 60 and 70; 4, older than 70
Gender	0, female; 1, male
Education	Education levels: 1, primary or below (reference group); 2, lower secondary; 3, upper secondary; 4, tertiary or above
City of residence	1, Beijing (reference group); 2, Shenyang; 3, Chengdu; 4, Nanjing; 5, Guangzhou
Income	Monthly income: 1, less than 1000 yuan (reference group); 2, between 1000 and 2000 yuan; 3, more than 2000 yuan
Medical insurance	1, urban resident basic medical insurance (URBMI) (reference group); 2, urban employee basic medical insurance (UEBMI); 3, new rural cooperative medical insurance (NRCM); 4, government insurance
Currently smoking	1 if smoking at the time of baseline survey, 0 otherwise
Currently during	1 if consuming alcohol at the time of baseline survey, 0 otherwise
Any physical exercise	1 if doing any physical exercise at the time of baseline survey, 0 otherwise
Diet control	1 if doing diet control at the time of baseline survey, 0 otherwise
Duration	Duration of diabetes. 1, less than five years (reference group); 2, between 5 and 10 years; 3, more than ten years
Heart disease	1 if heart disease, 0 otherwise
Hypertension	1 if hypertension, 0 otherwise
Dyslipidemia	1 if dyslipidemia, 0 otherwise
Stroke	1 if stroke, 0 otherwise
BMI	1 if BMI ≥ 24 at the time of baseline survey, 0 otherwise
HbA1c	1 if hemoglobin A1c < 6.5% at the time of baseline survey, 0 otherwise
FBS	1 if fasting blood sugar level <7 mmol/L at the time of baseline survey, 0 otherwise
Hypoglycemia	1 if reporting hypoglycemia at the time of baseline survey, 0 otherwise
SBP	1 if systolic blood pressure ≥ 140 at the time of baseline survey, 0 otherwise
DBP	1 if diastolic blood pressure ≥ 90 at the time of baseline survey, 0 otherwise
TC	1 if total cholesterol ≥ 5.2 mmol/L at the time of baseline survey, 0 otherwise
TG	1 if triglycerides ≥ 1.7 mmol/L at the time of baseline survey, 0 otherwise
HRQoL	1 if EQ-5D HRQoL ≥ 0.9 at the time of baseline survey, 0 otherwise

**Table 2:** Treatment therapies at baseline.

	Number of subjects	Proportion (%)	Cumulative proportion (%)
Metformin	203	10.67	10.67
Xiaoke Pill	233	12.24	22.91
Other TCMs	137	7.20	30.11
Gliclazide	128	6.73	36.84
Acarbose	110	5.78	42.62
Xiaoke Pill+	177	9.30	51.92
Glibenclamide	12	0.63	52.55
Others	903	47.45	100.00
Total	1903	100.00	

Note: we only kept those who have completed the baseline and all four follow-up surveys as well as two medical checks. Therapies in the category “others” are detailed in Appendix. TCMs refer to TCMs other than the Xiaoke Pill.

**Table 3:** Other observed plans on drug use.

Therapy	No. of cases	Prop.	Cum. prop.
Gliclazide + metformin	119	13.18	13.18
Metformin + acarbose	67	7.42	20.60
Other than these 15 drugs	57	6.31	26.91
Glipizide + metformin	50	5.54	32.45
Glimepiride + metformin	42	4.65	37.10
Glipizide	42	4.65	41.75
Gliquidone	36	3.99	45.74
Repaglinide	36	3.99	49.72
Gliclazide + acarbose	35	3.88	53.60
Gliclazide + metformin + acarbose	35	3.88	57.48
Repaglinide + metformin	29	3.21	60.69
Gliquidone + acarbose	26	2.88	63.57
Glimepiride	25	2.77	66.33
Glimepiride + acarbose	23	2.55	68.88
Glipizide + acarbose	20	2.21	71.10
Glimepiride + metformin + acarbose	18	1.99	73.09
Repaglinide + acarbose	17	1.88	74.97
Gliquidone + metformin	16	1.77	76.74
Metformin + TCMs	12	1.33	78.07
Acarbose + TCMs	9	1.00	79.07
Gliclazide + metformin + rosiglitazone	9	1.00	80.07
Rosiglitazone	9	1.00	81.06
Glibenclamide + metformin	8	0.89	81.95
Glipizide + metformin + acarbose	8	0.89	82.83
Nateglinide	8	0.89	83.72
Gliquidone + metformin + acarbose	7	0.78	84.50
Repaglinide + metformin + acarbose	7	0.78	85.27
Gliclazide + TCMs	6	0.66	85.94
Glimepiride + rosiglitazone	6	0.66	86.60
Glipizide + metformin + TCMs	6	0.66	87.26
Metformin + rosiglitazone	6	0.66	87.93
Pioglitazone	5	0.55	88.48
Gliclazide + metformin + TCMs	4	0.44	88.93
Metformin + pioglitazone	4	0.44	89.37
Phenformin	4	0.44	89.81
Gliclazide + rosiglitazone	3	0.33	90.14
Glimepiride + metformin + pioglitazone	3	0.33	90.48
Glipizide + gliclazide	3	0.33	90.81
Glipizide + gliclazide + metformin	3	0.33	91.14
Glipizide + TCMs	3	0.33	91.47
Metformin + rosiglitazone + acarbose	3	0.33	91.81
Repaglinide + rosiglitazone	3	0.33	92.14
Rosiglitazone + acarbose	3	0.33	92.47
Gliclazide + metformin + pioglitazone	2	0.22	92.69
Gliclazide + repaglinide	2	0.22	92.91
Glimepiride + metformin + pioglitazone + acarbose	2	0.22	93.13
Glimepiride + metformin + rosiglitazone	2	0.22	93.36
Glimepiride + pioglitazone	2	0.22	93.58
Glipizide + rosiglitazone	2	0.22	93.80
Gliquidone + acarbose + TCMs	2	0.22	94.02
Gliquidone + gliclazide	2	0.22	94.24
Gliquidone + rosiglitazone	2	0.22	94.46
Nateglinide + metformin	2	0.22	94.68
Pioglitazone + acarbose	2	0.22	94.91
Repaglinide + metformin + TCMs	2	0.22	95.13
Glibenclamide + acarbose	1	0.11	95.24
Glibenclamide + voglibose	1	0.11	95.35
Gliclazide + acarbose + TCMs	1	0.11	95.46
Gliclazide + glimepiride	1	0.11	95.57
Gliclazide + glimepiride + metformin	1	0.11	95.68
Gliclazide + metformin + rosiglitazone + acarbose	1	0.11	95.79
Gliclazide + metformin + rosiglitazone + acarbose + TCMs	1	0.11	95.90
Gliclazide + pioglitazone	1	0.11	96.01
Gliclazide + pioglitazone + acarbose	1	0.11	96.12
Gliclazide + rosiglitazone + acarbose	1	0.11	96.23
Gliclazide + rosiglitazone + voglibose	1	0.11	96.35
Glimepiride + metformin + TCMs	1	0.11	96.46
Glimepiride + nateglinide	1	0.11	96.57
Glimepiride + repaglinide	1	0.11	96.68
Glimepiride + rosiglitazone + acarbose	1	0.11	96.79
Glipizide + acarbose + TCMs	1	0.11	96.90
Glipizide + gliclazide + acarbose	1	0.11	97.01
Glipizide + glimepiride + acarbose	1	0.11	97.12
Glipizide + glimepiride + metformin + acarbose	1	0.11	97.23
Glipizide + gliquidone + metformin	1	0.11	97.34
Glipizide + gliquidone + metformin + rosiglitazone	1	0.11	97.45
Glipizide + metformin + pioglitazone	1	0.11	97.56
Glipizide + metformin + pioglitazone + acarbose	1	0.11	97.67
Glipizide + metformin + rosiglitazone	1	0.11	97.79
Glipizide + metformin + rosiglitazone + acarbose	1	0.11	97.90
Glipizide + pioglitazone	1	0.11	98.01
Glipizide + rosiglitazone + acarbose	1	0.11	98.12
Gliquidone + gliclazide + metformin	1	0.11	98.23
Gliquidone + metformin + acarbose + TCMs	1	0.11	98.34
Gliquidone + metformin + rosiglitazone	1	0.11	98.45
Gliquidone + metformin + TCMs	1	0.11	98.56
Gliquidone + nateglinide	1	0.11	98.67
Gliquidone + TCMs	1	0.11	98.78
Metformin + acarbose + TCMs	1	0.11	98.89
Metformin + phenformin + rosiglitazone	1	0.11	99.00
Metformin + pioglitazone + acarbose	1	0.11	99.11
Nateglinide + acarbose	1	0.11	99.22
Phenformin + acarbose	1	0.11	99.34
Repaglinide + acarbose + TCMs	1	0.11	99.45
Repaglinide + metformin + pioglitazone	1	0.11	99.56
Repaglinide + metformin + rosiglitazone	1	0.11	99.67
Repaglinide + pioglitazone	1	0.11	99.78
Repaglinide + TCMs	1	0.11	99.89
Rosiglitazone + TCMs	1	0.11	100.00
Total	903	100.00	

**Table 4:** Baseline characteristics (%).

	Metformin	Xiaoke Pill	Other TCMs	Glimepiride	Acarbose	Xiaoke Pill + others	Glibenclamide	Others	Total	ANOVA: *p* value
60 > age ≥ 50	25	31	26	20	15	25	17	25	25	0.06
70 >age ≥ 60	31	27	35	40	37	26	33	35	33	0.05
Age ≥ 70	22	20	31	30	34	24	8	28	27	0.03
Male	46	41	45	45	46	41	50	45	44	0.88
Lower secondary education	40	41	39	34	38	34	42	34	36	0.44
Upper secondary education	24	21	28	15	26	20	33	25	24	0.12
Tertiary education	14	16	7	9	17	16	0	13	13	0.07
Shenyang	33	42	74	17	18	10	33	12	23	0.00
Chengdu	24	27	6	16	26	33	25	19	21	0.00
Nanjing	16	8	4	53	12	5	42	24	19	0.00
Guangzhou	11	14	7	10	15	39	0	24	20	0.00
2000 > income ≥ 1000	49	37	53	31	31	28	58	38	38	0.00
Income ≥ 2000	31	33	20	23	51	46	0	39	36	0.00
UEBMI	65	64	69	41	72	63	58	65	64	0.00
NRCM	5	5	3	30	2	9	8	11	10	0.00
Govern. insur.	4	3	2	5	9	6	0	6	5	0.24
Currently smoking	25	21	27	16	19	18	33	19	20	0.18
Currently drinking	29	27	18	27	28	20	25	25	25	0.25
Any physical exercise	81	84	79	68	80	81	58	79	79	0.02
Diet control	89	85	84	88	93	92	92	91	90	0.03
10 > duration ≥ 5	19	20	24	35	19	29	42	28	26	0.00
Duration ≥ 10	17	17	34	16	15	24	17	29	24	0.00
Heart disease	18	21	40	20	25	16	17	19	21	0.00
Hypertension	53	35	55	48	64	46	8	51	49	0.00
Dyslipidemia	27	16	26	20	26	11	8	20	20	0.00
Stroke	11	5	16	13	10	5	0	7	8	0.00
Baseline BMI	67	54	59	70	55	47	42	58	58	0.00
Baseline HbA1c	42	53	29	37	51	46	33	33	39	0.00
Baseline FBS	47	61	31	42	59	54	33	39	45	0.00
Baseline hypoglycemia	12	9	9	10	8	9	8	13	11	0.35
Baseline SBP	44	33	44	54	39	38	50	39	40	0.01
Baseline DBP	33	27	28	37	18	27	42	23	26	0.00
Baseline TC	42	41	52	22	28	40	33	40	39	0.00
Baseline TG	51	39	46	39	33	38	50	41	41	0.04
Baseline HRQoL	47	52	46	45	55	53	50	46	48	0.46

Observations	203	233	137	128	110	177	12	903	1903	1903

Note: the last column includes significant levels derived from ANOVA tests regarding variable difference between different therapies.

**Table 5:** Unadjusted outcomes.

	HbA1c < 6.5%	Hypoglycemia	Endpoint HRQoL	Inpatient cost	Outpatient cost	OTC drug cost	Total cost
Metformin	0.33^b^	0.38^ab^	0.89^c^	4.22^c^	3.13^bc^	0.98^ab^	8.33^bcd^
	(0.03)	(0.05)	(0.01)	(0.91)	(0.34)	(0.13)	(1.01)
Xiaoke Pill	0.50^cd^	0.50^b^	0.90^c^	1.29^a^	1.96^a^	1.10^b^	4.35^a^
	(0.03)	(0.05)	(0.01)	(0.85)	(0.31)	(0.12)	(0.94)
Other TCMs	0.20^a^	0.72^c^	0.87^ab^	4.14^bc^	2.56^ab^	2.50	9.20^cd^
	(0.04)	(0.07)	(0.01)	(1.11)	(0.41)	(0.15)	(1.22)
Gliclazide	0.41^bc^	0.49^b^	0.86^a^	2.06^abc^	2.48^ab^	0.62^a^	5.15^a^
	(0.04)	(0.07)	(0.01)	(1.15)	(0.42)	(0.16)	(1.27)
Acarbose	0.45^cd^	0.33^ab^	0.89^bc^	4.36^bc^	5.94^d^	1.07^ab^	11.37^d^
	(0.05)	(0.07)	(0.01)	(1.24)	(0.46)	(0.17)	(1.37)
Xiaoke Pill+	0.54^d^	0.27^a^	0.88^abc^	1.43^ab^	3.82^c^	0.67^a^	5.92^ab^
	(0.04)	(0.06)	(0.01)	(0.98)	(0.36)	(0.14)	(1.08)
Glibenclamide	0.25^abc^	0.50^abc^	0.88^abc^	1.04^abc^	0.83^ab^	0.55^ab^	2.42^abc^
	(0.14)	(0.23)	(0.03)	(3.74)	(1.38)	(0.52)	(4.14)
Others	0.34^b^	0.39^b^	0.89^c^	3.16^abc^	5.57^d^	0.69^a^	9.42^cd^
	(0.02)	(0.03)	(0.00)	(0.43)	(0.16)	(0.06)	(0.48)

Observations	1903	1903	1903	1903	1903	1903	1903

Note: inpatient cost, outpatient cost, medication cost, and total cost are measured with the unit of 1000 RMB. Estimates sharing a letter in the group label are not significantly different at the 5% level.

**Table 6:** Adjusted outcomes: point estimates.

	HbA1c < 6.5%	Inci. of hypoglycemia	EQ-5D HRQoL	Inpatient cost	Outpatient cost	OTC drug cost	Total cost
Xiaoke Pill	0.12^*∗∗∗*^	0.07	0.00	−2.66^*∗∗*^	−0.52	−0.02	−3.20^*∗∗*^
	(0.04)	(0.07)	(0.01)	(1.27)	(0.39)	(0.16)	(1.37)
Other TCMs	0.03	0.13	−0.00	−1.26	0.45	0.70^*∗∗∗*^	−0.12
	(0.05)	(0.09)	(0.01)	(1.49)	(0.46)	(0.19)	(1.62)
Gliclazide	0.08	0.08	−0.02	−2.34	0.40	−0.10	−2.03
	(0.05)	(0.09)	(0.01)	(1.52)	(0.47)	(0.19)	(1.65)
Acarbose	0.07	0.05	−0.01	0.16	1.28^*∗∗∗*^	0.34^*∗*^	1.78
	(0.05)	(0.09)	(0.01)	(1.56)	(0.48)	(0.20)	(1.69)
Xiaoke Pill+	0.10^*∗∗*^	0.01	−0.02^*∗*^	−2.29^*∗*^	−0.03	0.05	−2.27
	(0.05)	(0.08)	(0.01)	(1.38)	(0.43)	(0.18)	(1.50)
Glibenclamide	−0.05	0.08	0.00	−3.75	−0.17	−0.50	−4.42
	(0.13)	(0.22)	(0.03)	(3.88)	(1.20)	(0.49)	(4.20)
Others	0.02	0.09	−0.00	−1.15	1.65^*∗∗∗*^	0.03	0.53
	(0.03)	(0.06)	(0.01)	(1.04)	(0.32)	(0.13)	(1.13)
60 > age ≥ 50	−0.05	0.01	0.00	0.41	1.28^*∗∗∗*^	−0.02	1.67
	(0.03)	(0.06)	(0.01)	(1.02)	(0.31)	(0.13)	(1.10)
70 > age ≥ 60	−0.11^*∗∗∗*^	−0.00	−0.01	2.18^*∗∗*^	1.03^*∗∗∗*^	0.14	3.36^*∗∗∗*^
	(0.03)	(0.06)	(0.01)	(1.03)	(0.32)	(0.13)	(1.12)
Age ≥ 70	−0.10^*∗∗∗*^	−0.03	−0.04^*∗∗∗*^	2.71^*∗∗*^	1.19^*∗∗∗*^	0.19	4.10^*∗∗∗*^
	(0.04)	(0.07)	(0.01)	(1.14)	(0.35)	(0.14)	(1.23)
Male	−0.00	−0.03	−0.00	0.64	−0.03	0.11	0.72
	(0.02)	(0.04)	(0.01)	(0.75)	(0.23)	(0.10)	(0.81)
Lower secondary education	0.01	−0.09^*∗*^	0.00	0.04	0.26	0.16	0.45
	(0.03)	(0.05)	(0.01)	(0.83)	(0.25)	(0.11)	(0.90)
Upper secondary education	−0.02	−0.03	0.00	0.53	0.80^*∗∗∗*^	0.56^*∗∗∗*^	1.89^*∗*^
	(0.03)	(0.05)	(0.01)	(0.94)	(0.29)	(0.12)	(1.01)
Tertiary education	0.01	−0.01	0.01	−0.11	0.46	0.34^*∗∗*^	0.69
	(0.04)	(0.07)	(0.01)	(1.16)	(0.36)	(0.15)	(1.26)
Shenyang	−0.04	0.56^*∗∗∗*^	−0.02^*∗*^	0.58	−6.94^*∗∗∗*^	1.93^*∗∗∗*^	−4.43^*∗∗∗*^
	(0.04)	(0.06)	(0.01)	(1.07)	(0.33)	(0.14)	(1.16)
Chengdu	0.24^*∗∗∗*^	0.01	0.01	0.08	−3.14^*∗∗∗*^	0.78^*∗∗∗*^	−2.28^*∗*^
	(0.04)	(0.06)	(0.01)	(1.09)	(0.34)	(0.14)	(1.18)
Nanjing	0.11^*∗∗∗*^	0.21^*∗∗∗*^	−0.00	0.11	−5.72^*∗∗∗*^	0.39^*∗∗∗*^	−5.22^*∗∗∗*^
	(0.04)	(0.07)	(0.01)	(1.15)	(0.35)	(0.15)	(1.25)
Guangzhou	0.19^*∗∗∗*^	0.05	−0.00	0.07	−4.19^*∗∗∗*^	0.42^*∗∗∗*^	−3.71^*∗∗∗*^
	(0.03)	(0.06)	(0.01)	(1.05)	(0.32)	(0.13)	(1.14)
2000 > income ≥ 1000	−0.03	−0.04	0.01	−0.11	0.62^*∗∗*^	0.01	0.52
	(0.03)	(0.05)	(0.01)	(0.89)	(0.27)	(0.11)	(0.97)
Income ≥ 2000	0.01	−0.04	0.02^*∗∗∗*^	−0.26	1.09^*∗∗∗*^	−0.09	0.75
	(0.03)	(0.06)	(0.01)	(1.01)	(0.31)	(0.13)	(1.09)
UEBMI	0.00	−0.03	0.00	0.58	0.13	−0.10	0.62
	(0.03)	(0.05)	(0.01)	(0.80)	(0.25)	(0.10)	(0.87)
NRCM	0.04	0.13^*∗*^	0.00	−1.37	−0.73^*∗*^	−0.13	−2.22
	(0.04)	(0.08)	(0.01)	(1.31)	(0.40)	(0.17)	(1.42)
Govern. insur.	0.00	−0.03	0.02	−2.12	−0.00	−0.15	−2.27
	(0.05)	(0.09)	(0.01)	(1.50)	(0.46)	(0.19)	(1.62)
Currently smoking	−0.03	0.02	−0.00	0.53	−0.33	−0.14	0.07
	(0.03)	(0.05)	(0.01)	(0.88)	(0.27)	(0.11)	(0.95)
Currently drinking	−0.03	−0.02	0.02^*∗∗*^	−0.28	−0.21	−0.17^*∗*^	−0.66
	(0.03)	(0.05)	(0.01)	(0.79)	(0.24)	(0.10)	(0.86)
Any physical exercise	−0.03	−0.08^*∗*^	0.03^*∗∗∗*^	−1.54^*∗∗*^	−0.10	0.05	−1.58^*∗*^
	(0.03)	(0.04)	(0.01)	(0.77)	(0.24)	(0.10)	(0.83)
Diet control	−0.03	0.03	−0.01	−0.64	0.64^*∗∗*^	−0.05	−0.05
	(0.03)	(0.06)	(0.01)	(1.00)	(0.31)	(0.13)	(1.09)
Duration ≥ 5	−0.01	0.03	−0.01^*∗∗*^	0.06	0.40^*∗*^	0.09	0.54
	(0.02)	(0.04)	(0.01)	(0.75)	(0.23)	(0.10)	(0.81)
Duration ≥ 10	−0.07^*∗∗∗*^	0.07	−0.01	1.34^*∗*^	0.44^*∗*^	0.42^*∗∗∗*^	2.20^*∗∗*^
	(0.03)	(0.05)	(0.01)	(0.79)	(0.24)	(0.10)	(0.86)
Heart disease	0.07^*∗∗∗*^	0.04	−0.01	0.53	0.87^*∗∗∗*^	0.40^*∗∗∗*^	1.80^*∗∗*^
	(0.03)	(0.05)	(0.01)	(0.79)	(0.24)	(0.10)	(0.86)
Hypertension	0.05^*∗∗*^	0.04	0.01^*∗*^	−0.51	0.93^*∗∗∗*^	−0.10	0.31
	(0.02)	(0.04)	(0.01)	(0.68)	(0.21)	(0.09)	(0.74)
Dyslipidemia	−0.02	0.01	0.00	0.07	0.57^*∗∗*^	0.28^*∗∗∗*^	0.92
	(0.03)	(0.05)	(0.01)	(0.80)	(0.25)	(0.10)	(0.87)
Stroke	−0.05	−0.04	−0.05^*∗∗∗*^	1.30	0.77^*∗∗*^	0.17	2.25^*∗*^
	(0.04)	(0.07)	(0.01)	(1.13)	(0.35)	(0.14)	(1.22)
Baseline BMI	−0.02	0.01	0.00	−0.47	0.08	0.01	−0.38
	(0.02)	(0.04)	(0.01)	(0.64)	(0.20)	(0.08)	(0.69)
Baseline HbA1c	0.26^*∗∗∗*^	0.03	0.00	−0.16	0.32	−0.01	0.15
	(0.02)	(0.04)	(0.01)	(0.73)	(0.22)	(0.09)	(0.79)
Baseline FBS	0.12^*∗∗∗*^	0.09^*∗∗*^	0.00	−0.23	−0.19	0.02	−0.40
	(0.02)	(0.04)	(0.01)	(0.70)	(0.22)	(0.09)	(0.76)
Baseline hypoglycemia	0.03	0.21^*∗∗∗*^	0.00	−0.88	0.09	0.08	−0.72
	(0.03)	(0.05)	(0.01)	(0.95)	(0.29)	(0.12)	(1.02)
Baseline SBP	−0.06^*∗∗∗*^	−0.06	0.01	0.03	−0.24	0.14	−0.07
	(0.02)	(0.04)	(0.01)	(0.74)	(0.23)	(0.09)	(0.81)
Baseline DBP	0.04	0.02	−0.02^*∗∗∗*^	0.53	−0.04	0.06	0.55
	(0.03)	(0.05)	(0.01)	(0.81)	(0.25)	(0.10)	(0.87)
Baseline TC	−0.03	0.02	−0.00	−0.68	−0.10	0.17^*∗∗*^	−0.61
	(0.02)	(0.04)	(0.01)	(0.65)	(0.20)	(0.08)	(0.70)
Baseline TG	0.03	−0.01	−0.00	1.06	−0.24	−0.09	0.74
	(0.02)	(0.04)	(0.01)	(0.65)	(0.20)	(0.08)	(0.70)
Baseline HRQoL	−0.02	−0.11^*∗∗∗*^	0.05^*∗∗∗*^	−1.35^*∗∗*^	−0.30	−0.05	−1.70^*∗∗*^
	(0.02)	(0.04)	(0.01)	(0.62)	(0.19)	(0.08)	(0.67)
Constant	0.24^*∗∗∗*^	0.24^*∗*^	0.86^*∗∗∗*^	4.45^*∗∗*^	4.56^*∗∗∗*^	−0.45	8.57^*∗∗∗*^
	(0.07)	(0.13)	(0.02)	(2.21)	(0.68)	(0.28)	(2.39)

Observations	1903	1903	1903	1903	1903	1903	1903

Note: metformin is the reference group. Significance level: ^*∗*^0.10, ^*∗∗*^0.05, and ^*∗∗∗*^0.01. Inpatient cost, outpatient cost, medication cost, and total cost are measured with the unit of 1000 RMB.

**Table 7:** Adjusted outcomes: predictive margins.

	HbA1c < 6.5%	Hypoglycemia	Endpoint HRQoL	Inpatient cost	Outpatient cost	OTC drug cost	Total cost
Metformin	0.33^a^	0.35^a^	0.89^ab^	4.28^b^	3.42^ab^	0.84^ab^	8.55^bcd^
	(0.03)	(0.05)	(0.01)	(0.93)	(0.29)	(0.12)	(1.00)
Xiaoke Pill	0.45^b^	0.42^a^	0.90^b^	1.63^a^	2.90^a^	0.81^ab^	5.34^a^
	(0.03)	(0.05)	(0.01)	(0.89)	(0.27)	(0.11)	(0.96)
Other TCMs	0.36^ab^	0.48^a^	0.89^ab^	3.02^ab^	3.87^bc^	1.54^c^	8.43^bcd^
	(0.04)	(0.07)	(0.01)	(1.19)	(0.37)	(0.15)	(1.29)
Gliclazide	0.41^ab^	0.43^a^	0.88^ab^	1.94^ab^	3.83^bc^	0.74^a^	6.52^abc^
	(0.04)	(0.07)	(0.01)	(1.20)	(0.37)	(0.15)	(1.30)
Acarbose	0.40^ab^	0.40^a^	0.88^ab^	4.44^ab^	4.70^cd^	1.18^bc^	10.33^d^
	(0.04)	(0.07)	(0.01)	(1.26)	(0.39)	(0.16)	(1.37)
Xiaoke Pill+	0.43^b^	0.36^a^	0.87^a^	1.99^ab^	3.40^ab^	0.89^ab^	6.28^ab^
	(0.03)	(0.06)	(0.01)	(1.01)	(0.31)	(0.13)	(1.09)
Glibenclamide	0.28^ab^	0.42^a^	0.89^ab^	0.53^ab^	3.26^abcd^	0.34^ab^	4.13^abcd^
	(0.12)	(0.22)	(0.03)	(3.77)	(1.16)	(0.48)	(4.09)
Others	0.36^a^	0.44^a^	0.89^b^	3.13^ab^	5.07^d^	0.87^ab^	9.07^cd^
	(0.01)	(0.03)	(0.00)	(0.45)	(0.14)	(0.06)	(0.48)

Observations	1903	1903	1903	1903	1903	1903	1903

Note: inpatient cost, outpatient cost, medication cost, and total cost are measured with the unit of 1000 RMB. When calculating the predictive margins, covariates including age, sex, education, household income, type of medical insurance, city of residence, diabetes-related morbidities including AMI, hypertension, dyslipidemia, and stroke, duration of diabetes, alcoholic use, smoking, physical exercise, diet control, BMI, blood glucose level, HbA1c, blood pressure, TCH, TG, and EQ-5D score are controlled. Estimates sharing a letter in the group label are not significantly different at the 5% level.

**Table 8:** Adjusted outcomes: predictive margins.

	HbA1c < 6.5%	Hypoglycemia	Endpoint HRQoL	Inpatient cost	Outpatient cost	OTC drug cost	Total cost
Metformin	0.25 A	0.25 A	0.90 B	2.73 A	3.36 A	0.60 BC	6.69 A
	(0.07)	(0.12)	(0.02)	(2.09)	(0.73)	(0.21)	(2.29)
Xiaoke Pill	0.42 B	0.37 A	0.89 B	2.59 A	3.80 A	0.24 AB	6.63 A
	(0.06)	(0.10)	(0.01)	(1.76)	(0.62)	(0.18)	(1.92)
Other TCMs	0.22 A	0.47 A	0.88 B	1.96 A	6.01 B	2.05	10.01 A
	(0.08)	(0.14)	(0.02)	(2.47)	(0.86)	(0.25)	(2.69)
Gliclazide	0.39 AB	0.26 A	0.90 B	0.21 A	4.06 AB	0.54 ABC	4.82 A
	(0.07)	(0.12)	(0.02)	(2.04)	(0.72)	(0.21)	(2.23)
Acarbose	0.46 B	0.24 A	0.87 AB	11.25 B	5.42 AB	1.08 C	17.75 B
	(0.08)	(0.14)	(0.02)	(2.39)	(0.84)	(0.24)	(2.61)
Xiaoke Pill+	0.33 AB	0.45 A	0.82 A	1.58 A	3.26 A	0.66 BC	5.49 A
	(0.07)	(0.12)	(0.02)	(2.02)	(0.71)	(0.21)	(2.21)
Glibenclamide	0.37 AB	0.44 A	0.90 AB	−0.25 AB	3.39 AB	−0.96 A	2.18 AB
	(0.25)	(0.45)	(0.06)	(7.59)	(2.66)	(0.77)	(8.29)
Others	0.36 AB	0.44 A	0.89 B	2.88 A	5.42 B	0.64 C	8.95 A
	(0.02)	(0.03)	(0.00)	(0.56)	(0.19)	(0.06)	(0.61)

Observations	878	878	878	878	878	878	878

Note: inpatient cost, outpatient cost, medication cost, and total cost are measured with the unit of 1000 RMB. When calculating the predictive margins, covariates including age, sex, education, household income, type of medical insurance, city of residence, diabetes-related morbidities including AMI, hypertension, dyslipidemia, and stroke, duration of diabetes, alcoholic use, smoking, physical exercise, diet control, BMI, blood glucose level, HbA1c, blood pressure, TCH, TG, and EQ-5D score are controlled. Estimates sharing a letter in the group label are not significantly different at the 5% level.

**Table 9:** Inverse-probability-weighted outcomes.

	HbA1c < 6.5%	Hypoglycemia	Endpoint HRQoL	Inpatient cost	Outpatient cost	OTC drug cost	Total cost
Metformin	0.36	0.38	0.90	4.09	3.21	0.85	8.15
	(0.04)	(0.05)	(0.01)	(1.02)	(0.25)	(0.09)	(1.16)
Xiaoke Pill	0.39	0.36	0.90	2.45	2.68	0.99	6.12
	(0.04)	(0.05)	(0.01)	(1.31)	(0.25)	(0.15)	(1.34)
Other TCMs	0.38	0.34	0.91	1.31	6.39	1.60	9.30
	(0.08)	(0.09)	(0.01)	(0.42)	(2.23)	(0.55)	(2.25)
Gliclazide	0.42	0.52	0.85	1.87	5.67	0.79	8.32
	(0.08)	(0.13)	(0.02)	(0.54)	(1.38)	(0.24)	(1.18)
Acarbose	0.39	0.43	0.88	4.58	4.73	1.35	10.66
	(0.05)	(0.08)	(0.01)	(1.57)	(0.48)	(0.42)	(1.75)
Xiaoke Pill+	0.39	0.41	0.87	1.26	3.94	1.01	6.21
	(0.05)	(0.10)	(0.02)	(0.40)	(0.42)	(0.27)	(0.70)
Others	0.35	0.43	0.89	3.01	5.04	0.88	8.93
	(0.02)	(0.03)	(0.00)	(0.41)	(0.15)	(0.09)	(0.45)

Observations	1903	1903	1903	1903	1903	1903	1903

Note: inpatient cost, outpatient cost, medication cost, and total cost are measured with the unit of 1000 RMB. Inverse probability weighting needs enough observations in each treatment arm during estimation, and we therefore merge glibenclamide into the category “others.” The predictive margins are calculated after multivariate regressions. When calculating the predictive margins, covariates including age, sex, education, household income, type of medical insurance, city of residence, diabetes-related morbidities including AMI, hypertension, dyslipidemia, and stroke, duration of diabetes, alcoholic use, smoking, physical exercise, diet control, BMI, blood glucose level, HbA1c, blood pressure, TCH, TG, and EQ-5D score are controlled.

**Table 10:** Baseline characteristics weighted by the inverse propensity score.

	Metformin	Xiaoke Pill	Other TCMs	Glimepiride	Acarbose	Xiaoke Pill + others	Others	ANOVA: + *p* value
60 > age ≥ 50	0.22	0.23	0.18	0.29	0.20	0.30	0.23	0.83
70 > age ≥ 60	0.33	0.29	0.27	0.19	0.35	0.29	0.34	0.17
Age ≥ 70	0.32	0.35	0.45	0.38	0.29	0.29	0.28	0.44
Male	0.42	0.45	0.50	0.44	0.51	0.44	0.43	0.92
Lower secondary education	0.34	0.30	0.34	0.29	0.41	0.37	0.35	0.75
Upper secondary education	0.24	0.27	0.26	0.40	0.27	0.23	0.23	0.80
Tertiary education	0.11	0.14	0.20	0.08	0.11	0.12	0.14	0.50
Shenyang	0.24	0.24	0.20	0.22	0.24	0.24	0.24	0.98
Chengdu	0.24	0.18	0.13	0.20	0.19	0.19	0.21	0.59
Nanjing	0.19	0.23	0.30	0.14	0.23	0.23	0.19	0.61
Guangzhou	0.18	0.21	0.22	0.13	0.14	0.16	0.20	0.55
2000 > income ≥ 1000	0.43	0.44	0.42	0.47	0.40	0.34	0.39	0.81
Income ≥ 2000	0.31	0.33	0.35	0.32	0.38	0.36	0.36	0.96
UEBMI	0.62	0.65	0.67	0.63	0.70	0.56	0.65	0.78
NRCM	0.11	0.08	0.12	0.09	0.05	0.14	0.10	0.80
Govern. insur.	0.06	0.04	0.03	0.03	0.04	0.04	0.05	0.88
Currently smoking	0.19	0.21	0.18	0.13	0.22	0.24	0.19	0.72
Currently drinking	0.20	0.30	0.29	0.37	0.24	0.31	0.25	0.43
Any physical exercise	0.76	0.81	0.91	0.79	0.82	0.79	0.79	0.01
Diet control	0.89	0.87	0.95	0.81	0.87	0.93	0.90	0.17
10 > duration ≥ 5	0.29	0.31	0.29	0.17	0.22	0.24	0.26	0.35
Duration ≥ 10	0.27	0.26	0.13	0.32	0.21	0.35	0.25	0.04
Heart disease	0.23	0.19	0.21	0.34	0.19	0.24	0.20	0.85
Hypertension	0.47	0.54	0.49	0.33	0.60	0.47	0.49	0.14
Dyslipidemia	0.20	0.22	0.17	0.12	0.24	0.21	0.20	0.54
Stroke	0.06	0.08	0.05	0.04	0.06	0.05	0.08	0.58
Baseline BMI	0.57	0.59	0.56	0.43	0.65	0.61	0.57	0.50
Baseline HbA1c	0.37	0.35	0.26	0.39	0.38	0.36	0.40	0.61
Baseline FBS	0.43	0.44	0.53	0.52	0.50	0.41	0.45	0.84
Baseline hypoglycemia	0.13	0.09	0.12	0.08	0.13	0.17	0.11	0.74
Baseline SBP	0.41	0.43	0.48	0.52	0.47	0.41	0.42	0.88
Baseline DBP	0.24	0.33	0.22	0.37	0.28	0.20	0.28	0.36
Baseline TC	0.38	0.44	0.40	0.49	0.32	0.44	0.39	0.63
Baseline TG	0.39	0.47	0.38	0.47	0.43	0.42	0.42	0.90
Baseline HRQoL	0.45	0.49	0.42	0.41	0.47	0.51	0.49	0.92

Note: observations are weighted by inverse propensity scores calculated from multinomial logistic regressions with regressors including demographic factors such as age and sex, socioeconomic factors such as education, household income, type of medical insurance, and city of residence, diabetes-related morbidities such as AMI, hypertension, dyslipidemia, and stroke, duration of diabetes, behavior factors such as alcohol use, smoking, physical exercise, and diet control, anthropometric and physiological indicators such as BMI, blood glucose level, HbA1c, blood pressure, TCH, TG, and HRQoL measured as EQ-5D score. The last column includes significant levels derived from ANOVA tests regarding the variable difference between treatment plans.

**Table 11:** Algorithm of double selection for variable selection.

(1) Select predictors of the outcome variable using adaptive lasso
(2) For each treatment arm {
Select predictors for treatment variable using adaptive lasso
}
(3) Take the covariates as the union of all predictors selected in steps 1 and 2
(4) Apply multivariate regression to the covariates selected

**Table 12:** Variable selected for post-LASSO OLS.

	HbA1c < 6.5%	Hypoglycemia	EQ-5D HRQoL	Inpatient cost	Outpatient cost	OTC drug cost	Total cost
60>age ≥ 50					Y		
70>age ≥ 60					Y		
Age ≥ 70			Y		Y		Y
Male							
Lower secondary education							
Upper secondary education					Y	Y	
Tertiary education							
Shenyang	Y	Y	Y	Y	Y	Y	Y
Chengdu	Y	Y	Y	Y	Y	Y	Y
Nanjing	Y	Y	Y	Y	Y	Y	Y
Guangzhou	Y	Y	Y	Y	Y	Y	Y
2000 > income ≥ 1000					Y		
Income ≥ 2000			Y		Y		
UEBMI							
NRCM	Y	Y	Y	Y	Y	Y	Y
Govern. insur.							
Currently smoking							
Currently drinking			Y				
Any physical exercise			Y				
Diet control							
10 > duration ≥ 5							
Duration ≥ 10	Y	Y	Y	Y	Y	Y	Y
Heart disease					Y	Y	
Hypertension	Y	Y	Y	Y	Y	Y	Y
Dyslipidemia							
Stroke			Y				
Baseline BMI							
Baseline HbA1c	Y	Y	Y	Y	Y	Y	Y
Baseline FBS	Y						
Baseline hypoglycemia							
Baseline SBP	Y						
Baseline DBP			Y				
Baseline TC	Y	Y	Y	Y	Y	Y	Y
Baseline TG							
Baseline HRQoL		Y	Y				
(60 > age ≥ 50) × (B/L HbA1c ctrl)							
(70 > age ≥ 60) × (B/L HbA1c ctrl)	Y						
(Age ≥ 70) × (B/L HbA1c ctrl)	Y	Y	Y	Y	Y	Y	Y
(Male) × (B/L HbA1c ctrl)							
(Lower secondary education) × (B/L HbA1c ctrl)							
(Upper secondary education) × (B/L HbA1c ctrl)	Y	Y	Y	Y	Y	Y	Y
(Tertiary education) × (B/L HbA1c ctrl)							
(Shenyang) × (B/L HbA1c ctrl)	Y						
(Chengdu) × (B/L HbA1c ctrl)					Y		
(Nanjing) × (B/L HbA1c ctrl)							
(Guangzhou) × (B/L HbA1c ctrl)							
(2000 > income ≥ 1000) × (B/L HbA1c ctrl)	Y	Y	Y	Y	Y	Y	Y
(Income ≥ 2000) × (B/L HbA1c ctrl)	Y	Y	Y	Y	Y	Y	Y
(UEBMI) × (B/L HbA1c ctrl)							
(NRCM) × (B/L HbA1c ctrl)							
(Govern. insur.) × (B/L HbA1c ctrl)							
(Currently smoking) × (B/L HbA1c ctrl)							
(Currently drinking) × (B/L HbA1c ctrl)							
(Any physical exercise) × (B/L HbA1c ctrl)							
(Diet control) × (B/L HbA1c ctrl)							
(10 > duration ≥ 5) × (B/L HbA1c ctrl)	Y	Y	Y	Y	Y	Y	Y
(Duration ≥ 10) × (B/L HbA1c ctrl)	Y						
(Heart disease) × (B/L HbA1c ctrl)							
(Hypertension) × (B/L HbA1c ctrl)							
(Dyslipidemia) × (B/L HbA1c ctrl)					Y		
(Stroke) × (B/L HbA1c ctrl)							
(Baseline BMI) × (B/L HbA1c ctrl)							
(Baseline FBS) × (B/L HbA1c ctrl)	Y	Y	Y	Y	Y	Y	Y
(Baseline hypoglycemia) × (B/L HbA1c ctrl)		Y					
(Baseline SBP) × (B/L HbA1c ctrl)							
(Baseline DBP) × (B/L HbA1c ctrl)							
(Baseline TC) × (B/L HbA1c ctrl)							
(Baseline TG) × (B/L HbA1c ctrl)							
(Baseline HRQoL) × (B/L HbA1c ctrl)					Y		

Note: B/L HbA1c ctrl is the abbreviation for baseline HbA1c control rate. The post-lasso linear regression is a two-step procedure where firstly confounding variables are selected using lasso and then they are used as controls in multivariate linear regression. To minimize the risk of overpenalization, variables selected for post-lasso regression are taken as the union of variables selected using both outcome and treatment arms as dependent variables of lasso. The choice of the tuning parameter of lasso is based on empirical BIC.

**Table 13:** Double selection.

	HbA1c < 6.5%	Hypoglycemia	Endpoint HRQoL	Inpatient cost	Outpatient cost	OTC drug cost	Total cost
Metformin	0.33^a^	0.35^a^	0.89^ab^	4.13^b^	3.46^ab^	0.86^a^	8.34^bc^
	(0.03)	(0.05)	(0.01)	(0.92)	(0.28)	(0.12)	(1.00)
Xiaoke Pill	0.44^b^	0.42^a^	0.90^b^	1.38^a^	2.86^a^	0.81^a^	5.04^a^
	(0.03)	(0.05)	(0.01)	(0.89)	(0.27)	(0.11)	(0.97)
Other TCMs	0.35^ab^	0.48^a^	0.89^ab^	3.34^ab^	3.80^bc^	1.53^b^	8.84^bc^
	(0.04)	(0.07)	(0.01)	(1.19)	(0.36)	(0.15)	(1.29)
Gliclazide	0.41^ab^	0.42^a^	0.87^ab^	2.16^ab^	3.82^bc^	0.80^a^	6.82^abc^
	(0.04)	(0.07)	(0.01)	(1.19)	(0.37)	(0.15)	(1.30)
Acarbose	0.40^ab^	0.39^a^	0.88^ab^	4.37^ab^	4.74^cd^	1.18^ab^	10.24^c^
	(0.04)	(0.07)	(0.01)	(1.26)	(0.39)	(0.16)	(1.37)
Xiaoke Pill+	0.44^b^	0.37^a^	0.87^a^	1.95^ab^	3.38^ab^	0.85^a^	5.95^ab^
	(0.03)	(0.06)	(0.01)	(1.01)	(0.31)	(0.13)	(1.09)
Glibenclamide	0.32^ab^	0.42^a^	0.89^ab^	0.95^ab^	3.26^abcd^	0.34^a^	4.07^abc^
	(0.12)	(0.22)	(0.03)	(3.77)	(1.16)	(0.48)	(4.10)
Others	0.36^ab^	0.44^a^	0.89^ab^	3.16^ab^	5.09^d^	0.87^a^	9.17^c^
	(0.01)	(0.03)	(0.00)	(0.45)	(0.14)	(0.06)	(0.48)

Observations	1903	1903	1903	1903	1903	1903	1903

Note: inpatient cost, outpatient cost, medication cost, and total cost are measured with the unit of 1000 RMB. The predictive margins are calculated after multivariate regressions. When calculating the predictive margins, covariates including age, sex, education, household income, type of medical insurance, city of residence, diabetes-related morbidities including AMI, hypertension, dyslipidemia, and stroke, duration of diabetes, alcoholic use, smoking, physical exercise, diet control, BMI, blood glucose level, HbA1c, blood pressure, TCH, TG, and EQ-5D score are controlled. Estimates sharing a letter in the group label are not significantly different at the 5% level.

## Data Availability

The data that support the findings of this study are available from the corresponding author upon reasonable request.

## Appendix

### B. On-Treatment Approach Treatment Effect

Table 8 and Figure 6 illustrate treatment effects based on the on-treatment approach, which admits a much smaller sample. No statistically significant difference among therapies in terms of control rate and adverse events was found, except that TCMs showed a lower control rate than the Xiaoke Pill and acarbose. Regarding costs, acarbose shows a higher total cost, which is statistically different from other plans. However, these differences should be read with caution as on-treatment analyses are based on a sample with a smaller size.

### C. Inverse Probability Weighting

Table 9 and Figure 7 show inverse-probability-weighted treatment effects, respectively, which are largely comparable with estimates from our multivariate linear regression. Both the control rate and the number of adverse events show no statistically significant difference among therapies. When cost is concerned, monotherapy or combination therapy using the Xiaoke Pill has the lowest costs, 6,200 and 6,200 RMB, respectively, per year. However, these values are not statistically different from the cost of metformin.

As indicated in Table 10, after propensity score weighting, almost all covariates became balanced among different therapies. For example, the baseline glycemic control rate (HbA1c < 6.5%) is similar among therapies and the difference is insignificant after weighting.

### D. Double Selection

To address causal treatment effect when making a variable selection, we use double selection [33] in the context of multiple treatment arms. The algorithm is described in Table 11.

In particular, we used lasso to select covariates from a large pool generated by including all control variables and their interactions, as shown in Table 12.

Table 13 and Figure 8 display estimates of multiple regressions after lasso selection. The results are very similar to the estimates from our multivariate regressions. The use of the Xiaoke Pill alone and its combination with other drugs has achieved better control rates, 44% against 33% of metformin. No significant difference is found in terms of hypoglycemia among different therapies, and the HRQoL difference is marginal. On average, the Xiaoke Pill costs each patient 5,040 RMB and metformin costs 8,340 RMB, respectively, per year, and the difference between the two is statistically different.
